The article "Utilizing Artificial Intelligence Among Patients With Diabetes: A Systematic Review and Meta-Analysis" was retracted in 2025. Reasons: fabricated or falsified data; unreliable results or conclusions; concerns about the data.

# Utilizing Artificial Intelligence Among Patients With Diabetes: A Systematic Review and Meta-Analysis

**DOI:** 10.7759/cureus.58713

**Published:** 2024-04-22

**Authors:** Abdullah Alhalafi, Saif M Alqahtani, Naif A Alqarni, Amal T Aljuaid, Ghade T Aljaber, Lama M Alshahrani, Hadeel Mushait, Partha​ A Nandi

**Affiliations:** 1 Department of Family and Community Medicine, University of Bisha, Bisha, SAU; 2 College of Medicine, University of Bisha, Bisha, SAU; 3 Department of Medicine, Batterjee Medical College, Aseer, SAU; 4 College of Medicine, King Khalid University, Abha, SAU

**Keywords:** ai models, north africa region, middle east, diabetes mellitus, artificial intelligence

## Abstract

Diabetes mellitus, a condition characterized by dysregulation of blood glucose levels, poses significant health challenges globally. This meta-analysis and systematic review aimed to evaluate the effectiveness of artificial intelligence (AI) in managing diabetes, underpinned by the Preferred Reporting Items for Systematic Reviews and Meta-Analyses (PRISMA) guidelines. The review scrutinized articles published between January 2019 and February 2024, sourced from six electronic databases: Web of Science, Google Scholar, PubMed, Cochrane Library, EMBASE, and MEDLINE, using keywords such as "Artificial intelligence use in medicine, Diabetes management, Health technology, Machine learning, Diabetic patients, AI applications, and Health informatics." The analysis revealed a notable variance in the prevalence of diabetes symptoms between patients managed with AI models and those receiving standard treatments or other machine learning models, with a risk ratio (RR) of 0.98 (95% CI: 0.88-1.08, I^2^ = 0%). Sub-group analyses, focusing on symptom detection and management, consistently showed outcomes favoring AI interventions, with RRs of 0.97 (95% CI: 0.87-1.08, I^2^ = 0%) for symptom detection and 0.97 (95% CI: 0.56-1.57, I^2^ = 0%) for management, respectively. The findings underscore the potential of AI in enhancing diabetes care, particularly in early disease detection and personalized lifestyle recommendations, addressing the significant health risks associated with diabetes, including increased morbidity and mortality. This study highlights the promising role of AI in revolutionizing diabetes management, advocating for its expanded use in healthcare settings to improve patient outcomes and optimize treatment efficacy.

## Introduction and background

Diabetes mellitus (DM) is a set of conditions brought on by abnormalities in the body's control over blood sugar levels. These conditions are brought on by the challenges encountered by the glucoregulatory system [1]. Persistent metabolic disease (diabetes) causes serious long-term harm to the kidneys, heart, blood vessels, nerves, and other organs. Most frequently, type 2 diabetes mellitus (T2DM) is linked to it [2].

The article "Utilizing Artificial Intelligence Among Patients With Diabetes: A Systematic Review and Meta-Analysis" was retracted in 2025. Reasons: fabricated or falsified data; unreliable results or conclusions; concerns about the data.

According to recent statistics, this illness is currently regarded as an epidemic and is becoming more widespread worldwide [3]. The overall prevalence of DM in Saudi Arabian citizens aged 30 and older is 24% [4]. Saudi Arabia currently ranks among the top 10 countries with the highest prevalence of diabetes. By 2030, it is expected to be among the top five countries with the highest prevalence of T2DM [5]. In the Middle East and North Africa, out of 73 million adults, approximately one in every six people has diabetes [5].

A sedentary lifestyle and an unhealthy diet are two of the main risk factors for T2DM. Additionally, some actions, like smoking and binge drinking, can increase the risk. The good news is that these risk factors are preventable. Changing for the better by eating a balanced diet and exercising to maintain a healthy weight can help lower the risk of T2DM [6].

Computer algorithms are used in the quickly evolving field of artificial intelligence (AI) to carry out tasks without the need for human intervention. Computers need structured data first, with each data point labeled or annotated in a language the algorithm can comprehend, to develop efficient AI algorithms. An algorithm's output is assessed to make sure it is accurate after it has been trained on a sufficient amount of labeled data. Observing and analyzing vast amounts of data, these AI algorithms are remarkably efficient at identifying patterns [7]. AI is being applied extensively in diabetes care in four key areas: screening for retinal disorders automatically, clinical advice and decision support, predicting risk for particular groups, and creating tools that allow patients to take care of their conditions on their own [8,9]. Based on this, the purpose of this study is to evaluate the usage of AI in diabetes management as well as the level of knowledge regarding its possible advantages.

## Review

Methodology

Article Search Strategy

Throughout the review process, the Preferred Reporting Items for Systematic Reviews and Meta-Analyses (PRISMA) guidelines were adhered to. To locate pertinent research, six electronic databases were searched: Web of Science, Google Scholar, PubMed, Cochrane Library, EMBASE, and MEDLINE [10]. This study focused on articles that had been published from January 2019 to February 2024. The keyword combinations used in the article search were "Artificial intelligence use in medicine, Diabetes management, Health technology, Machine learning, Diabetic patients, AI applications, and Health informatics."

The article "Utilizing Artificial Intelligence Among Patients With Diabetes: A Systematic Review and Meta-Analysis" was retracted in 2025. Reasons: fabricated or falsified data; unreliable results or conclusions; concerns about the data.

Eligibility, Data Extraction, and Management

A comparison of inclusion and exclusion criteria was used to confirm the eligibility of retrieved studies. The criteria for inclusion were that the articles should have been published in English since January 2019 and have undergone peer review. The population affected by diabetes or estimated to have the condition. There were no limitations on age, gender, or ethnicity; commercial, medical, or prototypes; wearable devices with AI, wearables that an individual can use without the assistance of clinical staff or in a hospital setting; and wearables that use noninvasive methods for diabetes analysis, empirical research examining diabetic blood glucose levels.

Articles excluded were those that were not peer-reviewed, published before January 2019, or not in English, involving patients unrelated to diabetes. Additionally, any research in which AI is not used as an intervention, not a wearable (such as a body-infused or artificial implant), research involving solely statistical methods for evaluating gathered information, sensors or tracking devices implanted within an individual's body, and wearable technology that requires appointments in a clinic or office.

Based on the stated criteria, independent screening and selection of the studies were conducted by two researchers. The PRISMA guidelines [10] were adhered to fully by the researcher and in case of disputes, discussion was conducted to reach a consensus. Finally, data was extracted and documented from the chosen studies.

Statistical Data Analysis

The software used in the analysis was Review Manager (RevMan) 5.4.1 (The Cochrane Collaboration, London, UK). In studies involving events, the metrics computed were risk ratio (RR), random effect (RE), standard error (SE), and 95% confidence intervals (CIs). The heterogeneity of the studies was measured using multivariate random-effects meta-regression that took into account both within and between study correlation. The I² values were categorized into four quartiles: low, low-to-moderate, moderate-to-high, and high heterogeneity, which ranged from 0% to <25%, 25% to <50%, 50% to <75%, and above 75%, respectively. The funnel plot asymmetry test and the quality of items' risk of bias assessment summary bar graph were used to quantify publication and item bias. All analyses were deemed statistically significant at the 0.05 level.

Results

Figure 1 shows a PRISMA diagram of the studies included in this analysis. A thorough search across several databases yielded 334 studies in total. Following the removal of duplicates, 112 articles were retained for further analysis. After 86 studies were excluded during the screening phase, 26 articles were selected for eligibility review. Eighteen of them were excluded because they didn't meet the predetermined requirements (inappropriate technique = 9, lack of full text = 9). Finally, eight studies were chosen for inclusion in the meta-analysis and systematic reviews.

The article "Utilizing Artificial Intelligence Among Patients With Diabetes: A Systematic Review and Meta-Analysis" was retracted in 2025. Reasons: fabricated or falsified data; unreliable results or conclusions; concerns about the data.

**Figure 1:** PRISMA flow diagram PRISMA: Preferred Reporting Items for Systematic Reviews and Meta-Analyses

Study Characteristics

All eight studies were carried out as randomized control trials in the English language. Furthermore, the investigated studies were conducted in a variety of countries and regions. These findings show that the studies vary significantly in terms of year, location, sample size, design, interventions, inclusions, and results. Table 1 displays these variations throughout each column.

**Table 1:** Study characteristics of the selected studies AI: artificial intelligence; ANNs: artificial neural networks; SVMs: support vector machines; DTs: decision tree algorithms

Author	Region	Sample size	Study design	Intervention	Inclusion	Outcomes/results
Chaki et al., 2022 [11]	Saudi Arabia	107	Randomized control trial systematic review and meta-analysis	Artificial intelligence and machine learning	Study design, intervention, and treatment	Recent developments in artificial intelligence and machine learning have made it feasible to identify and diagnose DM early using an automated method that is more accurate than a manual diagnosis.
Ansari et al., 2023 [12]	Pakistan	200	Randomized control trial	Artificial neural network models	Study design, intervention, and treatment	The results showed that the model with three hidden layers and Adam's optimization function was 98% accurate on the validation set. The utilization of diverse neurons in the hidden layers of the artificial neural network models enhanced their performance during training, thereby verifying the model's effectiveness and efficiency in assessing diabetes self-management practices according to the required data attributes.
Channa et al., 2023 [13]	America	3,160	Randomized control trial	AI and eye care providers	Study design, intervention, and treatment	Modeled risk differences of 90 per 100,000 were observed between groups receiving AI screening and the receiving eye care providers. Five years later, the AI-screened group had an estimated incidence of 1,535 vision loss per 100,000 people, while the group receiving eye care was estimated to have 1,625 vision loss per 100,000 people.
Bellemo et al., 2019 [14]	Zambia	13,099	Randomized control trial	AI and healthcare providers	Study design, intervention, and treatment	The detection of the prevalence of diabetic retinopathy that can be referred to and the correlations between the AI model, human graders, and systemic risk factors yielded similar results. Referable diabetic retinopathy was found to be associated with higher systolic blood pressure, longer duration of diabetes, and elevated glycated hemoglobin levels, as determined by both the AI model and human graders.
Elhadd et al., 2020 [15]	Qatar	13	Clinical randomized control trial	Machine learning artificial intelligence algorithms	Study design, intervention, and treatment	Extreme Gradient Boosting is an artificial intelligence machine learning algorithm that does a good job of anticipating both normal and hyperglycemic excursions. However, it is less effective at predicting hypoglycemia in patients who are fasting and are receiving multiple medications.
Alghamdi, 2023 [16]	Medina, Saudi Arabia	768	Randomized control trial	ANNs, SVMs, and DTs AI models	Study design, intervention, and treatment	Predicting diabetes complications with ANNs, SVMs, and DTs is in line with earlier research. The researchers demonstrated that the ANN models perform better than the other models in terms of sensitivity and accuracy, which is consistent with earlier research demonstrating the usefulness of ANNs as a method for predicting diabetes complications. However, a variety of factors, including the kind of outcome variable, the size and complexity of the dataset, and the requirement for interpretability, influence the choice of machine learning technique. Consequently, it's critical to select the best method based on the particular needs of the study.
Alfian et al., 2020 [17]	Korea	12	Randomized control trial; systematic review and meta-analysis	ANNs, SVMs, and DTs AI models	Study design, intervention, and treatment	These findings indicate that the recommended ANN-based blood glucose prediction model outperformed all other models. Our tests clearly showed that adding time-domain attributes to the input data improved the performance of most prediction models. The suggested prediction model will enable patients to track their blood glucose levels in the future. This will make it possible to create alerts that can be utilized to stop dangerous episodes of hyperglycemia or hypoglycemia.
Ellahham, 2020 [18]	United Arab Emirates	33,130	Retrospective cohort study randomized control trial	Artificial intelligence	Study design, intervention, and treatment	AI makes it possible to continuously and easily monitor a patient's biomarkers and symptoms remotely. Social media and online forums also improve patient participation in diabetes treatment. In the field of diabetes, technological advancements have improved resource efficiency. All of these clever technical changes have improved glycemic control by lowering glucose excursions, glycosylated hemoglobin, and fasting and postprandial glucose levels.

Risk of Bias Assessment

Figure 2 shows that most of the research was of very high quality, with little possibility of bias. A random sequence generator was used to prevent bias based on performance, detection, attrition, reporting, and selection. However, only a small proportion, 12.5% for each, of the research showed a high risk of detection bias and reporting bias, respectively.

The article "Utilizing Artificial Intelligence Among Patients With Diabetes: A Systematic Review and Meta-Analysis" was retracted in 2025. Reasons: fabricated or falsified data; unreliable results or conclusions; concerns about the data.

**Figure 2:** A summary of studies’ risk-of-bias of each item A risk-of-bias summary is provided based on an examination of the risk-of-bias items and the researcher's evaluations for each study. The red color denotes high risk, and the green color denotes low risk.

Meta-Analysis of the Outcome Assessment

Figures 3-5 show group and sub-group analysis of the use and potential benefits of AI in the management of diabetes. The overall prevalence of patients with diabetes symptoms differed significantly between the group treated using AI models and the comparator treatments (health professionals and other machine learning models) (RR: 0.98, 95% CI: 0.88-1.08, I^2^ = 0%; Figure 3). Sub-group analysis evaluated treatment outcomes based on diabetes (symptoms detection and management). Among the two sub-groups analyzed, there was a difference between the interventions used in treatments, all indicating a preference for AI treatment, as shown by the diamond markers. According to Figure 4, the symptoms detection group had (RR: 0.97, 95% CI: 0.87-1.08, I^2^ = 0%), and the management group had (RR: 0.97, 95% CI: 0.56-1.57, I^2^ = 0%; Figure 5).

**Figure 3:** Overall outcome AI models' forest plots for forecasting the identification and treatment of diabetes symptoms. The 95% CIs are shown by the horizontal lines. The effect value of a single study is represented by the square markers, and the total effect value of all the studies is represented by the diamond markers. The line of no effects is depicted by the vertical line. CI: confidence interval; df: degrees of freedom; p shows the significance of the test (p < 0.05 is considered significant)

**Figure 4:** Efficacy of AI in diabetes symptom detection AI models' forest plots for forecasting the identification and treatment of diabetes symptoms. The 95% CIs are shown by the horizontal lines. The effect value of a single study is represented by the square markers, and the total effect value of all the studies is represented by the diamond markers. The line of no effects is depicted by the vertical line. CI: confidence interval; df: degrees of freedom; p shows the significance of the test (p < 0.05 is considered significant)

**Figure 5:** Efficacy of AI in diabetes management AI models' forest plots for forecasting the identification and treatment of diabetes symptoms. The 95% CIs are shown by the horizontal lines. The effect value of a single study is represented by the square markers, and the total effect value of all the studies is represented by the diamond markers. The line of no effects is depicted by the vertical line. CI: confidence interval; df: degrees of freedom; p shows the significance of the test (p < 0.05 is considered significant)

Funnel Plots

Figure 6 shows a funnel plot that illustrates a symmetric distribution of effect sizes as a function of study precision with both sides having an equal number of studies. The symmetrical distribution of the sampled studies indicates a low risk of publication bias.

The article "Utilizing Artificial Intelligence Among Patients With Diabetes: A Systematic Review and Meta-Analysis" was retracted in 2025. Reasons: fabricated or falsified data; unreliable results or conclusions; concerns about the data.

**Figure 6:** Funnel plot depicting publication bias RR: relative risk; SE: standard error; X-axis: standard error; Y-axis: effect size

Discussion

Evaluating the application and possible advantages of AI in the treatment of diabetes was the goal of this meta-analysis and systematic review. The overall prevalence of patients with diabetes symptoms differed significantly between the group treated using the AI was found to have a better overall outcome compared to the group treated with other machine learning models and health professionals (RR: 0.98, 95% CI: 0.88-1.08, I^2^ = 0%). Complementing these results, a study by Chaki et al. discovered that developments in AI and machine learning have made it feasible to identify and diagnose DM early via an automated method that is more accurate than a manual diagnosis [11]. Further, according to these findings in a study by Ansari et al., the model utilizing Adam's optimization function and three hidden layers was found to be 98% accurate. Based on the required data attributes, the study's results improved the effectiveness and efficiency of artificial neural network (ANN) models in assessing diabetes self-management activities [12].

Among the two analyzed sub-groups, there was a difference between the interventions used for treatments, all of which favored AI treatment. In consistency with these findings, a study by Channa et al. modeled risk differences of 90 per 100,000 were observed between groups receiving treatment from eye care providers and the ones receiving AI screening. Five years later, the AI-screened group had an estimated incidence of 1,535 vision loss per 100,000 people, while the group receiving eye care was estimated to have 1,625 vision loss per 100,000 people. According to their study, if Americans adopted an autonomous AI-based screening strategy, they would experience vision loss after five years at a rate of 27,000 fewer than if they used an eye care professional. Due to various factors, the group that underwent AI screening experienced less vision loss five years later compared to the group that received medical eye care [13].

The article "Utilizing Artificial Intelligence Among Patients With Diabetes: A Systematic Review and Meta-Analysis" was retracted in 2025. Reasons: fabricated or falsified data; unreliable results or conclusions; concerns about the data.

However, the investigation of Bellemo et al. showed comparable outcomes when utilizing the AI model and human graders to determine the frequency of diabetic retinopathy that can be referred to as well as the relationships among systemic risk factors. Both the AI model and human graders identified elevated glycated hemoglobin levels, longer duration of diabetes, and higher systolic blood pressure as risk factors for referable diabetic retinopathy [14].

According to the study, the symptoms detection group had RR: 0.97, 95% CI: 0.87-1.08, I^2^ = 0%; and the management group had RR: 0.97, 95% CI: 0.56-1.57, I^2^ = 0% indicating AI was more effective in detection and management of diabetes. Aligned with these findings, a study by Elhadd et al. noted that machine learning AI algorithms such as Extreme Gradient Boosting (XGBoost) perform well in predicting normal and hyperglycemic excursions, but it is less predictive of hypoglycemia in patients receiving multiple medications while fasting [15].

Additionally, research carried out by Alghamdi supported these findings and revealed that ANN models perform better than the other models in terms of sensitivity and accuracy, thus demonstrating the usefulness of ANNs as a method for predicting diabetes complications. However, they saw that it is crucial to choose the most appropriate method based on the specific requirements of treatments [16]. More so, these findings in a study by Alfian et al. indicated that the recommended ANN-based blood glucose prediction model outperformed all other models. The study demonstrated that most prediction models performed better when time-domain attributes were added to the input data. It added that patients will be able to monitor their blood glucose levels in the future by utilizing the recommended prediction model. This will make it possible to create alerts that can be utilized to stop dangerous episodes of hyperglycemia or hypoglycemia [17]. Finally, as noted in a study by Ellahham, AI enables the continuous and convenient remote monitoring of a patient's biomarkers and symptoms. Social media and online forums also improve patient participation in diabetes treatment [18]. In diabetes, technological advancements have made resource usage more efficient. Together, these clever technical changes have improved glycemic control by lowering postprandial and fasting glucose levels, glucose excursions, and glycosylated hemoglobin.

The article "Utilizing Artificial Intelligence Among Patients With Diabetes: A Systematic Review and Meta-Analysis" was retracted in 2025. Reasons: fabricated or falsified data; unreliable results or conclusions; concerns about the data.

Limitations

This meta-analysis and systematic review face several limitations, including the potential for heterogeneity among AI models and study designs, which may affect results in comparability and generalizability. The narrow time frame of studies reviewed (from January 2019 to February 2024) might not fully capture the latest advancements in AI for diabetes management. Additionally, the reliance on studies published in English and indexed in selected databases could introduce language and publication bias, potentially overlooking relevant research. The focus on diabetes symptom prevalence as a primary outcome might also limit insights into other critical aspects of diabetes care facilitated by AI.

## Conclusions

Diabetes is linked to a number of side effects, such as mortality and morbidity. Diabetes needs to be treated as well as prevented, starting with an early diagnosis. As wearables and image visualization technologies develop, we think AI will become increasingly relevant in personalized lifestyle recommendations and diabetes care, especially in the area of disease detection. Therefore, future studies should be focused on areas that need to be advanced in AI in order to improve all dimensions of AI in the detection and management of diabetes.
